# Identification and Validation of Potential Biomarkers and Pathways for Idiopathic Pulmonary Fibrosis by Comprehensive Bioinformatics Analysis

**DOI:** 10.1155/2021/5545312

**Published:** 2021-07-04

**Authors:** Weibin Qian, Xinrui Cai, Qiuhai Qian, Xinying Zhang

**Affiliations:** ^1^Department of Lung Disease, Affiliated Hospital of Shandong University of Traditional Chinese Medicine, Jinan, 250011 Shandong, China; ^2^Department of Traditional Chinese Medicine, Shandong Academy of Occupational Health and Occupational Medicine, Shandong First Medical University & Shandong Academy of Medical Sciences, Jinan, 250062 Shandong, China; ^3^Department of Endocrinology, Affiliated Hospital of Shandong University of Traditional Chinese Medicine, Jinan, 250011 Shandong, China

## Abstract

**Objective:**

Idiopathic pulmonary fibrosis (IPF) is a chronic, progressive, irreversible, high-mortality lung disease, but its pathogenesis is still unclear. Our purpose was to explore potential genes and molecular mechanisms underlying IPF.

**Methods:**

IPF-related data were obtained from the GSE99621 dataset. Differentially expressed genes (DEGs) were identified between IPF and controls. Their biological functions were analyzed. The relationships between DEGs and microRNAs (miRNAs) were predicted. DEGs and pathways were validated in a microarray dataset. A protein-protein interaction (PPI) network was constructed based on these common DEGs. Western blot was used to validate hub genes in IPF cell models by western blot.

**Results:**

DEGs were identified for IPF than controls in the RNA-seq dataset. Functional enrichment analysis showed that these DEGs were mainly enriched in immune and inflammatory response, chemokine-mediated signaling pathway, cell adhesion, and other biological processes. In the miRNA-target network based on RNA-seq dataset, we found several miRNA targets among all DEGs, like RAB11FIP1, TGFBR3, and SPP1. We identified 304 upregulated genes and 282 downregulated genes in IPF compared to controls both in the microarray and RNA-seq datasets. These common DEGs were mainly involved in cell adhesion, extracellular matrix organization, oxidation-reduction process, and lung vasculature development. In the PPI network, 3 upregulated and 4 downregulated genes could be considered hub genes, which were confirmed in the IPF cell models.

**Conclusion:**

Our study identified several IPF-related DEGs that could become potential biomarkers for IPF. Large-scale multicentric studies are eagerly needed to confirm the utility of these biomarkers.

## 1. Introduction

Idiopathic pulmonary fibrosis (IPF) is a progressive, chronic, irreversible lung disease, characterized by an irreversible decline in lung function, progressive pulmonary scarring, and common interstitial pneumonia [1–3]. It affects more than 3 million people worldwide [4–7]. However, the prognosis of IPF remains poor, and the median survival time of patients is only 2-4 years [8, 9]. Thus, it emphasizes a need for a more complete understanding of the pathogenesis of IPF.

Long-term clinical work has shown that clarifying the pathogenesis of IPF helps to diagnose early disease, which is of great significance for the treatment of this disease, and has long-term clinical results to improve this fatal disease [9, 10]. However, it is still challenging to diagnose IPF in clinical work [11]. The clinical manifestations of IPF lack specificity, and the diagnosis needs to be combined with the detailed medical history of patients with multiple similar diseases [12, 13]. As the understanding of the disease deepens, biomarkers play an increasingly important role in the research and development of diseases [14, 15]. However, it is still difficult to reliably predict the course of IPF and the response to therapy for an individual patient [11]. There is a long way until biomarkers complete or substitute for the clinical and functional parameters currently available for IPF [16]. Only a very small number of DEGs have been found, and they are not consistent across all these studies [17]. Thus, further development into available markers and therapeutic targets is limited due to these inconsistent results [18]. Small sample sizes, different platforms, and different statistical methods are limiting factors that lead to inconsistent results [19]. To resolve this limitation, in this study, we comprehensively analyzed RNA-seq and microarray expression profiles of IPF from different platforms and validated hub genes in IPF cell models, which could lay the foundation for clinical research and IPF treatment.

miRNAs, a class of noncoding small RNAs, are involved in RNA silencing, posttranscriptional regulation, and other biological processes [20]. It has been confirmed that miRNAs play a critical role in the occurrence and development of various diseases, including IPF [21–23]. As an example, miR-92, miR-210, and miR-let-7d have been confirmed to be associated with IPF [24–26]. Therefore, in this study, differentially expressed genes (DEGs) in IPF were identified and miRNA-mediated regulatory network among all DEGs was constructed, which might shed novel light on molecular mechanisms of IPF progression.

## 2. Materials and Methods

### 2.1. Data Acquisition and Processing

The Gene Expression Omnibus (GEO) (http://www.ncbi.nlm.nih.gov/geo) is a public functional genomics data repository. Based on the filter criteria of keywords: IPF, organism: homo sapiens, and experiment type: expression profiling by high-throughput sequencing or expression profiling by array, two datasets GSE99621 and GSE110147 were included for this study. RNA-seq data of IPF were obtained from the GSE99621 dataset. This dataset contained 8 affected areas of the lung (IPF_S), 10 unaffected areas of the lung (IPF_N), and 8 healthy controls (N_CTL) on the GPL16791 platform [27]. The adapters were removed with Trimmomatic-0.38 and the localized Perl script was used to remove 5′ and 3′ low-quality bases (*Q* < 20), retaining sequences with *Q* > 20 bases above 90% and total length > 35 bp. The clean reads were mapped to the protein-coding gene sequence of Homo sapiens (assembly GRCh38.p12) using the HISAT2. Then, bedtools was utilized to calculate the number of reads and the RPKM expression value by a localized Perl script. After that, the GeneCluster3.0 was used for the systematic hierarchical clustering of samples. The principal component analysis (PCA) was then conducted. Microarray data of IPF were also retrieved from the GSE110147 dataset on the GPL6244 platform, including 22 IPF tissues and 11 normal lung tissues [28]. The flowchart of this study is shown in Figure 1.

### 2.2. Differentially Expressed Analysis

Differential expression analysis between the IPF_S, IPF_N, and N_CTL samples was performed using the limma package in R (http://bioconductor.org/packages/release/bioc/html/limma.html) [29]. Genes with adjusted *p* value ≤ 0.05 and fold change ≥ 1.5 were screened as upregulated genes. Meanwhile, those with adjusted *p* value ≤ 0.05 and fold change ≤ 1.5 were identified as downregulated genes.

### 2.3. Functional Enrichment Analysis

Gene Ontology (GO) and Kyoto Encyclopedia of Genes and Genomes (KEGG) enrichment analyses of DEGs were carried out by a functional annotation analysis tool online, Database for Annotation, Visualization and Integrated Discovery (DAVID; http://david.abcc.ncifcrf.gov/) [30]. In the biological processes, the gene expression heat maps most relevant to IPF were depicted. Terms with false discovery rate (FDR) < 0.05 were significantly enriched.

### 2.4. The miRNA-Target Network

The miRWalk 2.0 database was used to predict the relationships between DEGs and miRNAs. The miRWalk (http://mirwalk.uni-hd.de/) is a publicly available comprehensive resource that hosts predictive and experimentally validated miRNA-target interaction pairs. This database allows for possible miRNA binding site predictions within the complete sequence of all known genes in the three genomes (human, mouse and rat), including ten different prediction datasets [31]. We took the interactions between the three prediction sets of the TargetScan, miRDB and miRTarBase databases. Furthermore, a miRNA-target network was visualized using Cytoscape. Cytoscape is an open software platform for visualization and data integration of molecular interaction networks [32].

### 2.5. Common DEGs Both in RNA-seq and Microarray Datasets

Common DEGs were intersected between RNA-seq and microarray datasets. Furthermore, biological processes and pathways of these common DEGs were analyzed by GO and KEGG enrichment analyses. The peak map of DEGs was then built up.

### 2.6. Construction of a PPI Network

It is helpful to clarify the key mechanisms of disease development and reveal key cellular functions and biological processes by studying the interactions between transcripts or proteins. The data of BioGRID (http://www.thebiogrid.org) [33] and IntAct (http://www.ebi.ac.uk/intact) [34], two protein interaction databases, were integrated to find the interactions between common DEGs. Finally, a PPI network was visualized with Cytoscape software.

### 2.7. Cell Culture

Human normal lung and bronchus epithelial cell line BEAS-2B (CRL-9609, ATCC, USA) were grown in BEGM kit from Lonza (CC-3170; Basel, Switzerland) at 37°C in 5% CO_2_. BEAS-2B cells were treated with 0.5 ng/ml TGF-*β*1 for 48 h to construct an IPF cell model. The IPF model was validated by examining *α*-SMA, fibronectin, and Col I expression levels.

### 2.8. Western Blot

TGF-*β*1-induced BEAS-2B cells and controls were lysed by RIPA lysates (Beyotime, Shanghai, China). After the lysates were centrifuged at 12,000 × g for 20 min, the supernatant was harvested. The extracted protein was resolved by 10% SDS-PAGE and transferred onto PVDF membranes. Following blocking, the membranes were incubated with *α*-SMA (1 : 1000; ab108424, Abcam, USA), Fibronectin (1 : 1000; ab32419, Abcam), Col I (1 : 1000; ab255809, Abcam), GABARAPL1 (1 : 1000; ab229729, Abcam), GPX8 (1 : 1000; ab183664, Abcam), SGTA (1 : 1000; ab96571, Abcam), VCAM1 (1 : 1000; ab174279, Abcam), ARRB1 (1 : 1000; ab32099, Abcam), and GAPDH (1 : 1000; ab8245, Abcam), followed by secondary antibodies. The optical density of the bands was quantified using ImageJ software.

### 2.9. Statistical Analysis

All statistical analyses were carried out by R packages and GraphPad prism software. Each experiment was independently repeated at least three times. Data were presented as the mean ± standard deviation. Comparisons between two groups were presented by Student's *t*-test. *p* value < 0.05 indicated statistical significance.

## 3. Results

### 3.1. Upregulated and Downregulated Genes in IPF and Their Biological Functions

RNA-seq data of 8 IPF_S, 10 IPF_N, and 8 N_CTL samples were obtained from the GSE99621 dataset. Our hierarchical clustering analysis results showed that N_CTL samples were distinctly distinguished from IPF_S and IPF_N samples (Figure 2(a)). Several IPF_S and IPF_N samples were grouped into one category. In Figure 2(b), at the gene expression levels, there were significant correlations between the IPF_S, IPF_N, and N_CTL samples. Furthermore, PCA confirmed that N_CTL samples were different from the IPF_S and IPF_N samples (Figure 2(c)). With the cutoff of adjusted *p* < 0.05 and fold change ≥ 1.5, upregulated genes were screened between the IPF_S, IPF_N, and N_CTL samples (Figure 2(d)). We also identified downregulated genes with adjusted *p* < 0.05 and fold change ≤ 1.5 between the IPF_S, IPF_N, and N_CTL samples. Totally, 1224 genes were upregulated in the IPF_S than N_CTL samples, while 719 genes were downregulated in IPF_S compared to N_CTL samples. We explored potential biological functions of abnormally expressed genes between the IPF_S and N_CTL samples. Our data suggested that these upregulated genes were distinctly enriched in immune- or inflammatory-related pathways such as immune response, chemokine-mediated signaling pathway, inflammatory response, cell adhesion, extracellular matrix organization, monocyte chemotaxis, and lymphocyte chemotaxis (Figure 2(e)). In addition, these downregulated genes were mainly involved in IPF-related pathways such as oxidation-reduction process, angiogenesis, and cholesterol biosynthetic process (Figure 2(f)).

### 3.2. IPF-Related Upregulated Genes in Immune and Inflammatory Responses

Each stage of IPF is accompanied by innate or adaptive immune response [35]. Herein, we found that upregulated genes were mainly enriched in immune and inflammatory pathways. We further focused on which genes were involved in these pathways. As a result, chemokine (C-C motifs such as CCL-11, 13, 18, 21, 22, 24, 3, 3L1, 3L3, 4, 4L1, 4L2, 7, and 8 and C-X-C motifs such as CXCL10, 11, 12, 13, 14, 6, and 9) ligand family members and human leucocyte antigen (such as HLA-DOA, DOB, DPA1, DPB1, DQA1, DQB1, DQB2, DRA, DRB1, and DRB3) genes were significantly enriched in immune and inflammatory responses (Figure 3).

### 3.3. IPF-Related Upregulated Genes in Chemotaxis and Chemokine-Mediated Signaling Pathway

There is evidence that severity of IPF relies on chemotaxis [36].  Figure 4(a) showed all the upregulated genes enriched in chemotaxis and chemokine-mediated signaling pathway. Chemokine (C-C motifs such as CCL-11, 13, 18, 19, 21, 22, 24, 3, 3L1, 3L3, 4, 4L1, 4L2, 7, and 8 and C-X-C motifs such as CXCL10, 11, 12, 13, 6, and 9) ligand family members were distinctly enriched in chemotaxis and chemokine-mediated signaling pathway.

### 3.4. IPF-Related Genes in Pulmonary Fibrosis Pathway

We focused on the up- and downregulated genes enriched by pulmonary fibrosis pathway. As shown in Figure 4(b), SPARC, HPS3, SFTPD, SFTPC, SFTPA1, and SFTPA2 were involved in the pulmonary fibrosis pathway, indicating that abnormal expression of these genes could participate in the pulmonary fibrosis pathway.

### 3.5. Prediction of Up- and Downregulated Genes Regulated by miRNAs

Based on the miRWalk 2.0 database, we predicted the relationships between IPF-related DEGs and upstream miRNAs. The miRNA-target network for IPF was constructed (Figure 5). Our data showed that a DEG was often regulated by multiple miRNAs. For example, TGFBR3 was a target of hsa-let-7e-5p, hsa-let-7g-5p, hsa-let-7i-5p, hsa-miR-103a-3p, hsa-miR-107, hsa-miR-15b-5p, and hsa-miR-16-5p. RAB11FIP1 was regulated by hsa-miR-106a-5p, hsa-miR-106b-5p, hsa-miR-17-5p, hsa-miR-205-5p, hsa-miR-373-3p, hsa-miR-520a-3p, hsa-miR-520b, hsa-miR-520d-3p, hsa-miR-520e, and hsa-miR-93-5p.

### 3.6. Validation of DEGs and Their Biological Functions in IPF

To further validate DEGs in IPF, we comprehensively analyzed DEGs of IPF both in the microarray and RNA-seq datasets. As shown in Figure 6(a), 304 genes were upregulated in IPF_S compared to N_CTL both in the microarray and RNA-seq datasets. Furthermore, we found 282 downregulated genes in IPF_S compared to N_CTL both in the microarray and RNA-seq datasets. We further validated the biological functions enriched by these DEGs. In Figure 6(b), we listed the most significantly biological processes or pathways enriched by up- or downregulated genes, respectively. Our data confirmed that cell adhesion, extracellular matrix organization, collagen catabolic organization, collagen fibril organization, and extracellular matrix disassembly were significantly enriched by these upregulated genes. Moreover, we found that downregulated genes were most enriched in oxidation-reduction process and lung vasculature development. We gave an example of MMP7 expression in the IPF_S, IPF_N, and N_CTL samples (Figure 6(c)). We found the differences in the expression pattern of DEGs between the IPF_S and N_CTL samples in cell adhesion, extracellular matrix organization, oxidation-reduction process, and lung vasculature development (Figure 6(d)).

### 3.7. Construction of a PPI Network Based on Common DEGs in IPF

The PPI network was constructed to investigate the interactions between common DEGs both in the microarray and RNA-seq datasets (Figure 7). In the network, there were 227 nodes, including 122 upregulated and 105 downregulated genes. Nodes with degree ≥ 7 were considered hub genes, including GABARAPL1, GPX8, SGTA, VCAM1, ARRB1, SPP1, and HLA-B (Table 1).

### 3.8. miRNA-Target Network Based on Common DEGs in IPF

We further predicted the miRNAs of common DEGs both in the microarray and RNA-seq datasets. A miRNA-target network was established (Figure 8). We found that LDLR and RAB11FIP1 were regulated by most miRNAs. Both were upregulated in IPF_S compared to N_CTL.

### 3.9. Validation of Hub Genes in IPF Cell Models

TGF-*β*1-induced BEAS-2B cells were used to construct IPF cell models (Figure 9(a)). After verification, *α*-SMA, fibronectin, and Col I proteins were all highly expressed in TGF-*β*1-induced BEAS-2B cells than controls, suggesting that these IPF cell models were successfully constructed (*p* < 0.0001; Figures 9(b) and 9(c)). The hub genes were validated in TGF-*β*1-induced BEAS-2B cells by western blot. Our data confirmed that GABARAPL1, SGTA, and ARRB1 exhibited lower expression levels in IPF cells compared to controls (*p* < 0.0001; Figures 9(d) and 9(e)). GPX8 and VCAM1 were both downregulated in IPF cells than controls.

## 4. Discussion

In this study, we identified IPF-related DEGs (such as GABARAPL1, SGTA, ARRB1, GPX8, and VCAM1) and analyzed potential pathways (such as immune and inflammatory pathways) by comprehensively analyzing IPF-related RNA-seq and microarray datasets. Combining the PPI network, miRNA-target network, and functional enrichment analysis, we screened out potential biomarkers and their related regulatory mechanisms in IPF. These biomarkers might provide novel ideas and clues for further experimental research.

In this study, we analyzed DEGs between IPF_S and N_CTL. Functional enrichment analysis showed that upregulated genes in IPF_S were mainly enriched in immune response, chemokine-mediated signaling pathway, and cell adhesion and the like. Numerous molecules involved in immune response have been proposed as potential biomarkers for IPF [37]. For example, pyroptosis, a proinflammatory form of programmed cell death, mainly mediates the activation of caspase-1 through inflammasomes. A recent study has found that immunosuppressive molecule PD-L1 may trigger pyroptosis of pulmonary arterial smooth muscle cells, thereby accelerating pulmonary vascular fibrosis [38]. In addition, downregulated genes were mainly involved in oxidation-reduction process, angiogenesis, and cholesterol biosynthetic process and so on. It has been confirmed that reducing protein oxidation could reverse lung fibrosis [39]. Among all biological processes and pathways, we found that chemokine (C-C motif and C-X-C motif) ligand family genes were obviously associated with these significant biological processes, indicating that chemokine ligand family genes could play a key role in the processes of IPF, which was consistent with a previous study [40]. Also, a prospective case control study has found that chemokine ligand family member CCL18 is associated with IPF [41].

It has been well recognized that small sample sizes, different platforms, and different statistical methods could lead to inconsistent results [17, 42]. Therefore, in this study, we comprehensively analyzed DEGs between IPF_S and N_CTL both in the RNA-seq and microarray datasets. Our results showed that there are 304 upregulated genes and 282 downregulated genes in IPF_S compared to N_CTL both in the microarray and RNA-seq datasets. Functional enrichment analysis results revealed that these DEGs were mainly enriched in cell adhesion, extracellular matrix organization, oxidation-reduction process, and lung vasculature development. The PPI network showed that 3 upregulated including GPX8, VCAM1, and SPP1 and 4 downregulated genes including GABARAPL1, SGTA, ARRB1, and HLA-B could be considered hub genes for IPF. Among them, VCAM1 and TGFBR3 have been reported to be involved in the development of IPF. It has been confirmed that VCAM1 may mediate the adhesion of lymphocytes, monocytes, eosinophils, and basophils to vascular endothelium. Furthermore, it plays a key role in leukocyte-endothelial cell signal transduction. It is currently widely believed that VCAM1 is involved in the pathogenesis of atherosclerosis and can serve as a potential therapeutic target [43, 44]. More importantly, Agassandian et al. and other studies have shown that VCAM-1 can induce TGF-*β*1 expression upregulation and increase fibroblast expression in IPF [45]. Furthermore, GABARAPL1 may be involved in mediating the proliferation of endothelial progenitor cells, migration angiogenesis, and autophagy [46]. Methylated SGTA has been implicated in synovial fibroblast proliferation in patients with rheumatoid arthritis [47]. Based on the above findings, these hub genes might have potential effects in the pathogenesis of IPF, which require further research.

It has been confirmed that miRNA-mRNA interactions play a critical role in the development of IPF [48–50]. Here, we predicted the potential miRNA targets of all DEGs using the miRWalk 2.0 database. We found that DEGs were potential targets of many miRNAs, especially RAB11FIP1 and TGFBR3, indicating that the altered expression of these DEGs could be induced by miRNAs at the posttranscriptional level. For example, Rab11FIP1, a member of the large Rab GTPase family, has a regulatory role in the formation, targeting, and fusion of intracellular transport vesicles [51, 52]. As described in previous studies, Rab11FIP1 may play a vital role in several cancers such as breast cancer and cervical cancer [51, 52]. Otherwise, Hwang et al. believed that Rab coupling protein could activate epithelial-to-mesenchymal transition [53]. Interestingly, it has been proved that epithelial-to-mesenchymal transition is a key step in the development of IPF [54, 55]. Combining previous studies, Rab11FIP1 has the potential to become a potential biomarker for IPF.

Collectively, this study provided several novel draggable-target molecules for IPF by bioinformatics. The reliability of results for biological investigations was verified in IPF cell models. The consistent results between bioinformatics and biological investigation suggested convincing evidence that hub genes including GABARAPL1, SGTA, ARRB1, GPX8, and VCAM1 were abnormally expressed in IPF and could be utilized as a promising novel target for IPF treatment. However, there are several limitations in our study. First, although we validated hub genes in IPF cell models by western blot, their functions in IPF should be clarified. Second, although several pathways were identified for IPF, molecular experiments should be presented to prove more reliable evidence for the phenotypes and pathways underlying IPF. In conclusion, our study identified several IPF-related DEGs that could become potential biomarkers for IPF. Large-scale multicentric studies are eagerly needed to confirm the utility of these biomarkers in our future studies.

## 5. Conclusion

In this study, we comprehensively analyzed IPF-related DEGs and potential signaling pathways using the RNA-seq and microarray datasets. By combining the PPI network, miRNA-target network, and functional enrichment analysis, we identified potential biomarkers including GABARAPL1, SGTA, ARRB1, GPX8, and VCAM1 for IPF. Among them, GABARAPL1, SGTA, and ARRB1 exhibited lower expression levels in IPF while GPX8 and VCAM1 were both downregulated in IPF. These biomarkers might provide novel insights for further experimental research.

## Figures and Tables

**Figure 1:** The flowchart of this study.

**Figure 2:** Identification of DEGs and relevant signaling pathways for IPF using the GSE99621 RNA-seq dataset. (a) Hierarchical clustering analysis of 8 affected areas of the lung (IPF_S), 10 unaffected areas of the lung (IPF_N), and 8 healthy controls (N_CTL). (b) Volcano map and scatter plot showing the DEGs between IPF_S and N_CTL and between IPF_N and N_CTL. Red represents upregulated genes, and blue represents downregulated genes. (c) PCA analysis of 8 IPF_S, 10 IPF_N, and 8 N_CTL. (d) Venn diagram showing up- or downregulated genes between IPF_S and N_CTL and between IPF_N and N_CTL. (e) Functional enrichment analysis of upregulated genes. (f) Functional enrichment analysis of downregulated genes.

**Figure 3:** The difference in expression pattern of immune and inflammatory response-related DEGs in IPF_N, IPF_S, and N_CTL.

**Figure 4:** The difference in expression pattern of chemotaxis and chemokine-mediated signaling pathway- or pulmonary fibrosis-related DEGs in IPF_N, IPF_S, and N_CTL. (a) Chemotaxis and chemokine-mediated signaling pathway. (b) Pulmonary fibrosis.

**Figure 5:** miRNA-target network for IPF. The greater the degree, the larger the node. Red represents upregulated genes, green represents downregulated genes, and blue indicates miRNAs.

**Figure 6:** Identification of common DEGs and relevant biological processes or pathways for IPF both in the microarray and RNA-seq datasets. (a) Venn diagram showing the common DEGs for IPF_S both in the microarray and RNA-seq datasets. (b) Functional enrichment analysis of common up- or downregulated genes in IPF_S compared to N_CTL. (c) Gene peak map of MMP7. (d) The difference in expression pattern of cell adhesion-, extracellular matrix organization-, oxidation-reduction process-, and lung vasculature development-related DEGs in IPF_S and N_CTL.

**Figure 7:** The construction of protein-protein interaction network based on common DEGs both in the microarray and RNA-seq datasets. Red represents upregulated genes, and green represents downregulated genes.

**Figure 8:** miRNA-target network based on common DEGs both in the microarray and RNA-seq datasets. The greater the degree, the larger the node. Red represents upregulated genes, green represents downregulated genes, and blue indicates miRNAs.

**Figure 9:** Validation of hub genes in IPF cell models by western blot. (a) Construction of TGF-*β*1-induced IPF cell models. (b, c) Assessment of the expression of *α*-SMA, fibronectin, and Col I proteins in IPF cells. (d, e) Validation of the expression of GABARAPL1, SGTA, ARRB1, GPX8, and VCAM1 in IPF cells. ^∗∗∗∗^*p* < 0.0001.

**Table 1:** Hub genes in the PPI network.

Node	Degree	Up-/downregulation
GABARAPL1	12	Down
GPX8	12	Up
SGTA	11	Down
VCAM1	10	Up
ARRB1	9	Down
SPP1	7	Up
HLA-B	7	Down

## Data Availability

The datasets analyzed during the current study are available from the corresponding author on reasonable request.

## Abbreviations

IPF: Idiopathic pulmonary fibrosis
DEGs: Differentially expressed genes
PPI network: Protein interaction network
PCA: Principal component analysis
DAVID: Database for Annotation, Visualization and Integrated Discovery
GO: Gene Ontology
KEGG: Kyoto Encyclopedia of Genes and Genomes.
